This article has been retracted.

# Advanced multimodal imaging of solid thyroid lesions with artificial intelligence-optimized B-mode, elastography, and contrast-enhanced ultrasonography parametric and with perfusion imaging: Initial results

**DOI:** 10.3233/CH-239102

**Published:** 2023-07-18

**Authors:** E.M. Jung, C. Stroszczynski, F. Jung

**Affiliations:** Institute of Diagnostic Radiology and Interdisciplinary Ultrasound Department, University Hospital, Regensburg, Germany; Institute of Biotechnology, Brandenburg University of Technology, Senftenberg, Germany

**Keywords:** Thyroid lesions, multimodal ultrasound, artificial intelligence (AI), UMA-elastography, contrast enhanced ultrasonography (CEUS), parametric-perfusion analysis

## Abstract

Goal of the study was the assessment of AI-assisted diagnosis of solid thyroid foci with multimodal modern ultrasound imaging. 50 patients (26–81 years, 54.7±13.1 years) were included in the study. Multimodal ultrasound imaging by means of B-mode with linear probe (4–12 MHz) with option of automated documentation of findings by means of AI, with supplementary Ultra MicroAngiography (UMA) was used. Macrovascularisation was assessed by dynamic contrast ultrasonography (CEUS) with parametric evaluation and perfusion analysis, and microvascularization was assessed by combined strain and shear wave elastography on a novel high-performance ultrasound system (Resona R9/Mindray) by an experienced examiner with independent reading. The evaluation was performed according to TI-RADS III-V.

The volume of the thyroid lobes on both sides averaged 39 ml±5 ml (27 to 69 ml). The 13 cases of histologically confirmed thyroid carcinomas (8 papillary, 2 medullary, 2 microfollicular, 1 anaplastic CA) with a mean size of 15 mm±6 mm (9–21 mm) were correctly evaluated by TI-RADS V on the basis of irregular shape, induration > 2.5 m/s or > 30kPA and striking wash-out kinetics. Tumor lymph nodes could only be correctly detected preoperatively in one case of medullary carcinoma according to the surgical findings, based on irregular vascularization with UMA in roundish shape with cortex > 4 mm, transverse diameter up to 11 mm. In 25 cases of inhomogeneous nodular goiter an evaluation with TI-RADS III was performed in 31 cases, in 4 cases with incomplete marginal contour, partial marginal vascularization with UMA and partial wash out with indurations up to 2.5 m/s 30 kPA an evaluation with TI-RADS IV and surgical excision for nodular goiter. In 12 cases regressive nodular changes without relevant malignancy criteria resulted in nodular goiter, with focal changes up to 1.5 cm in diameter, classified as requiring control with TI-RADS III. There were no relevant changes in findings in the controls after 6 months. From the AI tool, the 20/25 goiter nodes were assessed as TI-RADS III, 7/12 adenomas, 5 goiter nodes, and 5 adenomas as TI-RADS IV, 5/13 carcinomas as TI-RADS IV, and 8/13 carcinomas as TI-RADS V.

Multimodal ultrasound diagnostics supported by AI has a high diagnostic potential for the evaluation of solid thyroid lesions and standardizes the reporting with digital representative image documentation. CEUS perfusion and modern elastography techniques allow targeted follow-up of TI-RADS III findings.

## 1 Introduction

Ultrasound is the most widely used imaging modality and provides a variety of diagnostic options in the evaluation of thyroid glands and decisions about interventional procedures or surgery [1–3]. Thus, in the hands of experienced examiners, nodular changes can be further clarified, cysts and complicated cysts can be assessed, changes in macro- and microvascularization can be detected, and malignant tumors can also be identified at an early stage [1–4].

The criteria of the fundamental B-scan leading to an assessment of benignity or malignancy of thyroid lesions have been summarized in the TI-RADS classification [5]. Irregular echo-inhomogeneous foci with microcalcifications that may have microcalcifications and are also irregularly vascularized are particularly suspicious for malignancy. The size and size dynamics of malignancy-suspect foci also play an important role [1–3, 5, 6].

Due to increasingly improving ultrasound technology with high-resolution multifrequency probes, cystic as well as complicated cystic lesions and tumor foci can be assessed with modern ultrasound even at small sizes of less than 1 cm in diameter [1–6]. Initial artificial intelligence (AI) approaches are being used to attempt to detect suspicious thyroid foci, size them, and digitally document criteria for classification according to TI-RADS in a standardized manner [7–10].

With ultrasound elastography in strain technique with manual compression or automated in shear wave technique, tissue compaction can be displayed in false colors and assessed semiquantitatively or evaluated quantitatively [11–13]. This is particularly successful when both techniques are performed in parallel.

New vascular ultrasound techniques can then be used as an additional criterion of sonomorphology to investigate the extent to which the vascular pattern of solid tumor foci is regular or irregular. Nevertheless, Doppler techniques are limited with respect to the detection of low flows and even the smallest vessels. If hemodynamic parameters are adjusted to very low values, a large number of artifacts may occur, making valid assessment difficult. Here, new high-resolution techniques of low-angle-dependent ultrasound microangiography (UMA) seem promising [14].

Down to the capillary region, contrast-enhanced ultrasonography (CEUS) can be used to dynamically detect tumor microvascularization. With CEUS, wash-in and wash-out dynamics can be assessed and perfusion analysis can also be performed. However, it is not possible to capture the hemodynamics of flow changes with standard techniques of CEUS. Then, parametric false color display and perfusion evaluation with time intensity curve analysis (TIC analysis) with different perfusion parameters can help [4, 15, 16].

It remains to be investigated to what extent it is possible to use the V-flow also for the assessment of thyroid lesions. In order to assess the histopathology of thyroid lesions with absolute certainty, it is useful to compare it to the surgical result. In this pilot study, multimodal ultrasound examinations of the thyroid gland in solid nodular changes prior to planned surgery will be demonstrated for the first time in the combination of UMA, combined elastography techniques and CEUS parametric and perfusion analysis. To demonstrate criteria for modified evaluation of TI-RADS III-V lesions with CEUS.

## 2 Materials and methods

Inclusion criterion was preparation for immediate surgery by indication through interdisciplinary case conferences with endocrinologic, nuclear medicine, and surgical evaluation.

All examinations with ultrasound contrast medium sonography (CEUS) were performed after written consent. The evaluation of the examinations was performed retrospectively with the approval of the local ethics committee ((20-2122-104).). The examinations were requested after preliminary examinations by special outpatient clinics with the question of the assessment of solid thyroid lesions that had been noticed in out-of-town preliminary examinations. An evaluation according to TI-RADS III-V had to be performed and it had to be decided to what extent a histological clarification was necessary or whether a follow-up should be performed.

All examinations were performed by an experienced investigator (more than 3000 examinations per year, over more than 20 years) using a linear multifrequency probe (L 4–12 MHz) on high-performance ultrasound equipment (Resona R9, Mindray, China) with digital image documentation in PACS. This allowed independent subsequent evaluation by experienced readers. According to the predefined scheme of an artificial intelligence (AI) image evaluation program, both thyroid lobes were measured in longitudinal and transverse axis with length, depth and width, the volume was calculated, the echogenicity was evaluated as homogeneous, discrete inhomogeneous or inhomogeneous and the echo pattern was judged as echo-complex or echo-normal.

The ultrasound elastography techniques available in parallel mode as strain or shear wave elastography were used to assess compaction of thyroid tissue and solid foci. The pulsatile region of a carotid artery was bypassed as much as possible to avoid artifacts. Image quality could be assessed automatically, optimally with 5 green stars. False colors informed about homogeneous or inhomogeneous compaction. Measured values over individually adjusted regions of interests (ROI) could be recorded in m/s or kPA, with values > 2.5 m/s or > 30 kPA considered suspicious for possible malignant lesions.

Detectable solid lesions were also measured by AI in three planes, and the rim contour was bypassed for volumetric detection. Then, marginal contour had to be assessed as regular, lobulated or irregular, rim as complete or incomplete, or absent, growth axis, parallel or directed in depth, shape as oval or roundish, and possible macro- or microcalcifications and entered into a predetermined scheme. After localization of the suspicious lesion, the evaluation according to TI-RADS III-V was then color-coded in a final scheme with topogram. This then also considers a possible tumor vascularization, as irregular malignancy-suspicious, or as regular marginal benign.

UMA (Ultra MicroAngiography) was used to assess the vascularization of tumor foci in as much detail as possible with velocity ranges < 10 cm/s. Vascular patterns were recorded dynamically in short cine loops up to 10 s. This also captured possible conspicuous lymph nodes with regular benign vascularization from the hilus or malignancy-typical from the margin.

Macrovascularization of thyroid lobes and foci was classified as normal, enhanced, or decreased, and that of foci as regular or irregular. Color-coded duplex sonography (CCDS), HR flow with glazing flow, and UMA were used for this purpose.

The criterion for benign findings was a regular vascular pattern, especially a marginal vascularization, for example in adenomas. Irregular vascularization was considered suspicious for malignancy. This was then additionally investigated with contrast medium sonography (CEUS) to determine the extent to which irregular arterial hypervascularization with delayed wash out occurs, which is evaluated as a malignancy criterion.

Contrast ultrasonography (CEUS) after bolus administration of 1 to 1.5 ml of sulphuhexafluoride microbubbles (SonoVue®/BRACCO) with 10 ml of saline solution cubital, if possible, was used to assess dynamic microvascularization of the suspicious solid lesions. When possible, cine loops of incipient arterial vascularization after 10 to 15 s up to one minute were then evaluated parametrically and by time intensity curve (TIC) using the High-End Devices internal perfusion program. Regions of interest (ROI) were individually matched, in the center, at the edge of the lesion to be assessed compared with surrounding thyroid tissue. Parametric color maps were fitted to the corresponding perfusion parameters such as time to peak (TTP), peak, mean transit time (mTT), wash in area under the curve (wash in AUC) and tabulated at the end.

## 3 Results

50 cases (26–81 years, mean age: 43±7 years) were examined with multimodal imaging consisting of B-mode, UMA, elastography and CEUS with parametric and perfusion analysis with good to very good image quality in all cases, according to the internal evaluation mode especially in the shear wave elastography technique with clearly > 85% or 5 green stars.

The volume of the thyroid lobes on both sides averaged 39 ml±5 ml (27 to 69 ml).

All echo-poor, irregularly vascularized, inhomogeneously indurated lesion > 1 cm were identified as highly suspicious for malignancy with early wash out kinetics and were also confirmed surgically.

The 13 cases of histologically confirmed thyroid carcinoma (8 papillary, 2 medullary, 2 microfollicular, 1 anaplastic carcinoma) with a mean size of 15 mm±6 mm (9–21 mm) were correctly evaluated by TI-RADS IV based on irregular shape, induration > 2.5 m/s or > 30kPA and appositional wash-out kinetics using CEUS (TI-RADS V) (Figs. 1, 2).

**Fig. 1:** Ultrasound elastography, simultaneous evaluation by strain and shear wave elastography of a suspicious malignant thyroid tumor (TI-RADS IV). Lower stiffness of the center (blue) and irregular higher stiffness at the margin (yellow and red) with values up to 2.5 m/s.

**Fig. 2:** CEUS after bolus injection of 1.5 ml contrast agent (SonoVue®) with irregular microvascularization of a malignant thyroid tumor (TI-RADS V). Color coded perfusion imaging with evaluation of different perfusion parameters (PKI, AT, AUC, WiAUC). Dynamic detection of the tumor microvascularization using time intensity curve (TIC) evaluation from the early arterial phase after 15 sec up to 1 minute.

Tumor lymph nodes could be correctly detected preoperatively only in one case of medullary carcinoma according to the surgical findings, based on irregular vascularization with UMA in roundish shape with cortex > 4 mm with a transverse diameter up to 11 mm.

In 25 cases of inhomogeneous nodular goiter, evaluation with TI-RADS III was performed in 31 cases, evaluation with TI-RADS IV was performed in 4 cases with incomplete marginal contour, partial marginal vascularization with UMA and partial wash out with indurations up to 2.5 m/s or 30 kPA, and surgical excision was performed for nodular goiter (Fig. 3).

**Fig. 3:** Case of a small intracystic papillary thyroid cancer (TI-RADS IV). Irregular vascularization detected by CCDS and UMA in different color modalities (upper line). Irregular stiffness detected by simultaneous mode of strain and shear wave elastography (left down). Characterization by B-Mode criteria using AI (right down).

In 12 cases of adenomas with diameters of 1.7 to 3.5 cm, mean 26 cm±0.5 cm, nodular goiter resulted in proportionately regressive nodular changes. Only in 7/12 cases a typical echo-poor rim and a typical rim vascularization were found. In 5 cases, the rim was incomplete. Contrast ultrasonography (CEUS) also showed a partial central wash out in these cases with but preserved marginal vascularization and elastography revealed partial induration up to 2.5 m/s or 30 kPA an assessment with TI-RADS III or IV rating (Fig. 4).

**Fig. 4:** Echoinhomogeneous thyroid tumor with some criteria for a benign lesion but also inhomogeneous center of the tumor. Automatically detection using AI options (Smart Thyroid) for measurements of the tumor size and also for finally evolution of the tumor morphology considering TI-RADS III. Histopathology after surgery was a benign tumor with central necrosis.

Using the AI tool, the 20 of 25 goiter nodes were evaluated as TI-RADS III, 7 of 12 adenomas, 5 goiter nodes and 5 adenomas as TI-RADS IV, 5 of 13 carcinomas as TI-RADS IV and 8 of 13 carcinomas as TI-RADS V. Microcalcification as a definite malignancy criterion was automatically detected in 5 of 13 malignancies, an echo-poor irregular echo structure in all cases, and in intracystic tumors in 2 cases. The shape was irregular in all cases, proportionately lobulated, but oriented in depth in only 8 of 13 cases. Of the 25 struma nodules evaluated as possibly also malignant, partial necrosis and inhomogeneous microvascularization with also induration on elastography occurred in all cases (Fig. 5).

**Fig. 5:** Multimodality ultrasound diagnosis of medullary thyroid carcinoma (TI-RADS V) with inhomogeneous compaction in strain and shear wave elastography (top left), with irregular micro-vascularization with CEUS (top right, bottom left) and documentation and evaluation with AI tools bottom right.

For 37 patients both classifications were identical. From the 12 cases, histologically classified as TI-RADS V, 11 were also classified as TI-RADS V by the AI-based diagnosis.

Of the 13 remaining cases in which there were discrepancies between the two methods, 12 were histologically confirmed grade 3 carcinoma. Using AI-based diagnostic they were classified at least one grade higher by AI (*n* = 12, including 2 two grades higher) and in one case a histologically confirmed as TI-RADS V case one grade lower (Fig. 6).

**Fig. 6:** Classification of the thyroid carcinoma according to the histological (in blue) as well as to the AI-based findings (in red) for the 50 patients.

## 4 Discussion

The basis for classification according to TI-RADS remains high-resolution B-scan sonography and, in addition, color Doppler [5–7]. Elastography and contrast medium sonography (CEUS) are also increasingly used [4, 12, 13, 15]. The aim is to assess thyroid lesions as accurately as possible in terms of benignity and malignancy.

In addition to shape and size, echogenicity, marginal contour, rim, depth, micro- or macrocalcification and possible pathological lymph nodes play an important role in the evaluation of solid lesions as benign or malignant. At least 1% of all cases of solid thyroid nodules in the general population are malignant. The task of modern multimodal ultrasound diagnostics is the earliest possible and reliable detection and, if necessary, a targeted biopsy with the help of ultrasound.

Using artificial intelligence (AI) approaches, suspicious lesions are first detected, then outlined and longitudinal diameter and transverse diameter measured. Then the characterization can be entered into a predefined scheme, adapted to the criteria of TI-RADS [8–10]. Then, finally, an evaluation is made and color-coded a localization in the scheme. Red-coded lesions to be histologically confirmed are then urgently entered in the topogram as TI-RADS IV or V findings.

Another approach of this pilot study was to examine to what extent an irregular vascular pattern typical for malignant lesions can already be detected with the technique of Ultra Micro Angiography (UMA). This could then be another criterion in the evaluation of unclear non-cystic lesion. At least the results indicate that in parts a differentiation between rather regular flow in benign thyroid lesions and irregular vascular pattern in malignant lesions is successful. With adaptation to lower flow fractions < 10 cm/s, artifacts of color Doppler such as aliasing, pulsations, zero flow detection at 90 degrees of egg sound angle can be overcome with UMA. One can even have a direction coded flow display or a subtraction image without background information.

Another approach of the new multimodal ultrasound diagnostics is the parallel examination with strain and shear wave elastography. This not only increases the comparability in TI-RADS III lesions, but also the assessment of malignancy-suspicious foci with increased tissue compaction with measured values > 2.5 cm/s or > 30 kPA [4, 11–13].

Contrast sonography can be used to demonstrate irregular neovascularization typical of malignant lesions and an early wash out [4, 15, 16]. This can be visualized parametrically with false colors, red for a fast hypervascularization, followed by orange and yellow, then already less strong with green and delayed with blue and violet. If regions of interest (ROI) are selected in the center, in the margin and the normal SD tissue, benign lesions are characterized by a regular margin pattern without early wash out.

In malignant lesions, hypovascularization can be detected as a delayed increase by time intensity curve (TIC) already within the first minute after contrast bolus administration. Or irregular hypervascularization with early onset wash out may occur. With the new integrated perfusion software, wash in and wash out kinetics of CEUS can be mapped parametrically within less than 1 min for the different perfusion parameters, such as time to peak (TTP), peak, mean transit time (mTT), wash in area under the curve (AUC) [4]. In addition, based on the TIC analysis in curve form, the values are also presented finally in table form.

The initial results of this study suggest that multimodality ultrasound imaging with AI may be helpful in differentiating TI-RADS III lesions from TI-RADS IV or V findings. Vividly, the extent of suspicious thyroid lesions can succeed with the AI tool. Based on shape, contour, echogenicity, vascularization and depth, criteria for a benign or malignant lesion can be documented automatically. Nevertheless, the evaluation of microcalcifications may then require manual re-evaluation.

If the results of the elastography measurements are also taken into account with regard to the possible tissue compaction of the tumors, additional criteria for malignancy can be obtained at high values. CEUS is helpful if wash out kinetics is to reveal the possible malignancy of individual foci in struma multinodosa [4–16]. Adenomas may show a central wash out in parts with persistent marginal vascularization. Carcinomas show a wash out from the margin. Intracystic tumors like papilloma’s are irregularly vascularized and become distinguishable from complicated septate cysts with sedimentation by CEUS [4, 15, 16, 24, 25]. Already by optimizing for low flow, UMA can help to make the marginal vascularization in adenomas more recognizable.

Critically, ultrasound alone can never differentiate carcinoma from inhomogeneous struma nodules in all cases. Thus, it is understandable that a wide variability of malignancy from 15 to 85% may be present in TI-RADS IV findings [5, 17, 24–26]. Thus, in case of doubt, histologic confirmation becomes necessary, especially when scintigraphy is not directional in small suspicious tumor foci [18, 19]. Also CEUS perfusion imaging could be a very important appositional tool for detection small intra-cystic tumors, characterization of small malignant tumor and differentiation TI-RADS III, IV, and V lesions [4, 20–27].

Nevertheless, the new multimodal ultrasound modalities offer the possibility of early detection of malignant foci. Multicenter evaluation is needed to evaluate the possibility of additional AI in terms of differentiation from TI-RADS III to TI-RADS V.
